RETRACTED

# Operating Room Planning for Emergency Surgery: Optimization in Multiobjective Modeling and Management from the Latest Developments in Computational Intelligence Techniques

**DOI:** 10.1155/2022/2290644

**Published:** 2022-02-17

**Authors:** Qiqian Li, Yali Liu, Esra Sipahi Döngül, Yufen Yang, Xiaoyuan Ruan, Wegayehu Enbeyle

**Affiliations:** ^1^The Seventh Affiliated Hospital of Southern Medical University, Guangzhou, Guangdong, China; ^2^The Sixth Affiliated Hospital of Sun Yat-Sen University, Guangzhou, Guangdong, China; ^3^Aksaray University, Faculty of Health Sciences, Department of Social Work, Aksaray, Turkey; ^4^Shenzhen University General Hospital, Shenzhen, Guangdong, China; ^5^The Eighth Affiliated Hospital of Sun Yat-Sen University, Guangzhou, Guangdong, China; ^6^Department of Statistics, Mizan-Tepi University, Tepi, Ethiopia

## Abstract

This study presents an optimization approach for scheduling the operation room for emergency surgeries, considering the priority of surgeries. This optimization model aims to minimize the costs associated with elective and emergency surgeries and maximize the number of scheduled surgeries. In this study, surgeon assistants to perform each surgery are considered in order to achieve the goals. Since the time of each surgery varies according to the conditions of the patient, this parameter is considered as an uncertain one, and a robust optimization method is applied to deal with uncertainty. To demonstrate the effectiveness of the proposed method, a case study in one of the East Asian hospitals is presented and analyzed using GAMS software. Moreover, hybrid simulation and gray wolf optimization algorithm (GWO) have been implemented to solve the optimization model in different scenarios. The results show that increasing the risk parameters in the robust optimization model will increase the system costs. Moreover, in case of uncertainty, the solutions obtained from the GWO simulation method are on average 73.75% better than the solutions obtained from the GWO algorithm.

## 1. Introduction

Living a healthy life and looking for solutions to health problems are some of the priorities of mankind in every age. The development of health sciences is made possible by the development of environmental impacts. Although medical science is perceived as a whole in itself, it is possible to see that it actually benefits from many disciplines when looking at the subject in detail. Although basic sciences such as physics, chemistry, and biology are leading the way, the solution proposals put forward by management and information systems, which have developed rapidly since the middle of the last century, have enabled these systems to be integrated into health sciences as well as social works. Social workers around the world serve as the primary professional leaders of an influential community centres movement [1].

RETRACTED

The field of medical social work is mainly aimed at solving urgent crises. In hospitals with a lot of patient turnover, social workers have to perform very fast and effective interventions. Therefore, working in this field requires special skills.

In recent decades, health and treatment costs have been increased, and the operating room is one of the most important areas in the hospital that needs regular management due to its high potential for cost savings [2]. Operating rooms are one of the most expensive and fundamental resources of a hospital. Therefore, poor scheduling may lead to periods of unemployment, overwork, delay in surgery, or cancellation of surgery, which results in additional costs and a lack of income for the hospital [3].

Despite the multiplication of costs in the field of health and the increase in the number of hospitals, increasing services of health systems have not been able to meet the growing demand [4]. Moreover, the most important challenges of health systems are the increasing demand for surgical services, random service times, limited access to resources, and patient-surgeon compatibility [5, 6]. Accordingly, operating room scheduling plays a crucial role in the operating room management.

In this study, a two-objective mathematical model for elective and emergency surgeries is examined by considering the priority of emergency patients over selected patients and assigning surgeon assistants to each surgery. Since the time of each surgery cannot be predicted, the uncertainty is considered for this parameter, and a robust optimization method is used to deal with uncertainty. The optimization method, which is one of the issues of interest to management sciences, comes to the aid of health and social service management at this point.

In this research, given the above and the sensitivity of operating room scheduling, an attempt has been made to present a model with the following innovations:

  Providing a two-objective mixed-integer model for scheduling the operating room, which includes (1) minimizing surgical costs, including the cost of shifting and the cost of not performing emergency surgery due to the operating room being not empty and (2) maximizing the number of surgeries performed
  Simultaneous consideration of surgery of emergency patients and selected patients
  Optimization of the mathematical model by considering the priority of emergency surgeries over selected surgeries
  Assigning a surgeon's assistant for each surgery
  Optimization of uncertainty problem by considering the surgical time parameter
  Providing a robust optimization method to deal with uncertainty in the studded problem
  Proposing a novel solution method based on the simulation and gray wolf optimization algorithm

The rest of the study is as follows: In Section 2, the studies conducted in this field are reviewed. In Section 3, the proposed operating room scheduling model is presented, and then, in Section 4, the uncertainty conditions for the surgical time parameter are applied and a robust optimization method to deal with the uncertainty is proposed. In Section 5, the results of solving the certain model as well as solving the uncertain model for different levels of conservatism are presented and compared, and in Section 6, the conclusion and future directions of the research are presented.

RETRACTED

## 2. Literature Review

The scheduling problem has been used in the manufacturing industry for many years but has recently come to the attention of many service industries, including the healthcare systems. The first research on operating room planning began in 1953 with Adair [7]. Surgeons believed that if enough space and assistance were available, surgeries can be increased by up to 50%. In the 1970s, Dal Ceilo [8] proposed a study of idle times in the operation room. In 1984, Charnetski [9] conducted one of the first studies of reducing idle time in healthcare systems.

Some researches in this field have examined the effect of patient preference and surgical timing on operating room planning in the context of social works. Min and Yih [2] examined a scheduling problem in which patients had different priorities and the facility capacity for a selective surgery was limited; in this way, when capacity is available, patients are selected with a higher priority than the waiting list and placed on a schedule. Abedini et al. [10] proposed a multistep approach to assigning surgeries to operating rooms and a priority scheduling rule. This rule categorizes surgeries based on their priority, type of surgery, and time, and their use reduces unemployment time, reduces the number of operating rooms required, and reduces the number of operating room startups.

Admission of emergency patients is an important issue for operating rooms, which can lead to delays throughout the system if resources are inadequate. Erdem et al. [11] proposed a model for rescheduling selected patients as soon as emergency patients arrived, intending to examine the overwork costs of the operating room and postanesthesia unit, the costs of delaying elective surgeries, and the costs of not admitting emergency patients. In a study by Lamiri et al. [12], a stochastic model for operating room planning is presented with two types of surgery requests (elective and emergency) in which emergency patient admission is random. In another study by these researchers [10], they examined an uncertain model for scheduling selective surgeries, considering the demand uncertainty for emergency surgeries.

RETRACTED

One of the critical points in scheduling emergency surgeries is scheduling them as quickly as possible because delaying them may increase the risk. Essen et al. [13] examined emergency surgeries in one of the operating rooms of choice. In this study, emergency patients undergo surgery as soon as an elective surgery is completed. Reserving operating room capacity as soon as an emergency patient arrives is a common way to maximize responsiveness. Bhattacharyya et al. investigated a case in which an operating room was reserved only for essential surgeries, and additional surgeries could be performed if an unreserved room was not available.

Equipment plays a crucial role in hospitals, mainly operating rooms, and their lack or unavailability may lead to surgical arrests as well as the death of patients. Therefore, planning and scheduling hospital equipment is essential, especially if the equipment is special or of great importance [12]. Therefore, some researchers have examined the issue of operating room scheduling by considering the required resources and equipment.

Beds are a scarce resource in the intensive care unit, and patients' random demand for these beds, as well as incidental service time, makes resource management a difficult issue. In a study using a simulation model, Seung-Chul et al. [14] evaluated different bed reservation schemes because they considered reserving some beds for the exclusive use of selected patients as one way to minimize canceled surgeries.

Roland et al. conducted a study considering the limitations of human resources and considering their preferences and the limitations of the volume of reusable materials and equipment with the aim of minimizing the costs due to overtime and operating room use. According to Latorre-Núñez et al. [3], in operating room scheduling, each surgery requires a specific combination of human resources, equipment and materials, and a bed to resuscitate the patient, and the timing should be such that in addition to scheduled surgeries, emergency surgeries that may occur during the day should also be considered. Silva et al. [15] modeled surgical scheduling using specialized human resources and social workers based on their skills as well as staff time window with the aim of maximizing the use of operating rooms. Molina-Pariente et al. [16] presented a model for solving the problem of operating room planning and scheduling in which the effect of the number of surgeons on surgical teams and the dependence of surgical time on their experience and skills were examined.

RETRACTED

Xiang [17] considered that operating room scheduling is generally a multiobjective problem. Next, they provided a meta-heuristic approach to solve the proposed multiobjective scheduling problems. Saadouli et al. [18] proposed a stochastic optimization and simulation approach for scheduling operating rooms and resuscitation beds with the aim of minimizing the maximum operating time and the total waiting time of each operating room. The effect of allowing the patient to be resuscitated in the operating room when the resuscitation bed is not available was investigated by Augusto et al.

The problem of resource uncertainty often coincides with the uncertainty of patient admission. For example, the arrival of emergency patients may be accompanied by complaints of the surgeon's absence for surgery and the unavailability of an operating room, which can lead to delays in elective surgeries [16]. Therefore, some researchers have examined operating room scheduling issues with uncertainty in mind. Persson and Persson [17] examined operating room planning, taking into account uncertainties in inpatient admission requests and surgical timing. Addis et al. [19] examined the issue of selecting a set of patients from the waiting list of selected patients and allocating them to available operating rooms. For each patient, the maximum waiting time and uncertainty during surgery are considered, and new patients' entry in their research is examined.

Liu et al. [20] studied surgical scheduling by simultaneously examining surgery priorities and operating room scheduling decisions. Considering the uncertainty at the time of surgery, they presented a robust model for minimizing surgical time, which reduced the surgical time by considering scenarios compared to definitive scheduling methods. Kroer et al. [21] examined the planning of operating rooms for a hospital in Denmark, in which each surgery must be assigned to a specific operating room, as well as surgery for a specific time in order to minimize overtime and use capacity. Nouaouri et al. [22] considered the uncertainty of inpatient admission and surgery time. They solved the problem by assuming a limited number of surgeons and operating rooms and with the aim of maximizing the number of surgeries performed in operating rooms. Khaniyev et al. [23] have dealt with operating room scheduling in case of surgery duration uncertainty. In this study, in which scheduling is done for only one day, first, a mathematical model is developed, and then, an innovative algorithm is introduced. Rahimi and Gandomi [24] provide a comprehensive overview of operating room scheduling. In this study, various optimization models and solution methods are introduced, and then, the importance of uncertainty in this issue is emphasized. Lin and Li [25] have solved the problem of operating room scheduling with meta-heuristic methods. In this study, a modified mathematical model is provided to optimize operating room costs as well as increase operating room utilization. The artificial bee colony (ABC) algorithm has also been used to optimize this mathematical model. The results show that for a number of surgeries between 40 and 100, the ABC algorithm can provide the optimal solution in a short time.

RETRACTED

As the literature shows, in many studies, selective surgeries have been examined in the operating room scheduling problem, and the arrival of emergency patients has been ignored. However, the arrival of emergency patients is an unavoidable issue, and not paying attention to emergency surgery cases may have life-threatening risks for patients. Uncertainty in surgical timing is also one of the issues that have been investigated in quantitative research if the timing of surgeries is not predictable and can only be estimated by examining similar previous surgeries, which is based on the specific characteristics of each surgery cannot be invoked. Moreover, having a surgeon's assistant with the surgeon for each surgery can lead to improvements in surgery time, unemployment time, overtime time and thus reduce surgery costs, as well as increase the quality of surgery and patient satisfaction. This issue, despite its importance, needs further study and research.

Considering the mentioned cases, despite their importance, has not been studied in a comprehensive study in previous researches. Accordingly, the purpose of this study is to provide a model to examine these research gaps in order to increase patient satisfaction.

## 3. Problem Statement

In this research, the efficiency of the proposed model of one of the Asian hospitals is studied. According to operating room officials, in hospitals, in addition to specialized operating rooms located in each ward, a number of operating rooms for surgeries that do not require specialized equipment exist in each ward. In this study, the number of operating rooms in the hospital is four, and the different types of surgeries performed in these rooms are 4.

In this research, to solve the multiobjective model, the LP-metric method is used in order to minimize the relative deviations of the goals from their optimal value. Moreover, the time of surgery is unpredictable due to the fact that it is affected by several factors. It is considered as an uncertainty parameter, and a robust optimization method is used to deal with uncertainty.

RETRACTED

The notations and symbols used in the proposed mathematical programming model are defined in the following.

### 3.1. Indices

 
*i*: selected patient index
 
*h*: emergency patient index
 
*j*: index of type of surgery
 
*r*: index of operating room
 
*t*: index of time period
 
*a*: index of collection of surgeon assistants

### 3.2. Parameters

 
*Bp*: capacity of the postoperative care unit (resuscitation beds) along the scheduling horizon
 
*Brt*: capacity of operating room
 
*Bat*: assistant surgeon a working time
 
*C*_*jtt′*_: the cost of postponing an elective surgery of type *j* scheduled for time *t*′ to time *t*
   *git*: binary parameter and equal to 1 if the patient's surgery *i* is scheduled for period *t*; 0 otherwise
 
*H*: number of emergency patients requesting surgery
 
*I*: the number of selected patients whose surgery is scheduled on the time horizon
 
*J*: the number of types of surgeries that can be performed with facilities
 
*m*_*ij*_: 1 if the selected patient *i* requests a type *j* surgery; 0 otherwise
 
*m′*_*hj*_: 1 if the emergency patient *h* requests a type *j* surgery; 0 otherwise
 
*R*: number of operating rooms
 
*O*_*j*_: the expected time for a type *j* surgery
 
*r*_*j*_: the cost of not performing type *j* emergency surgery on time
 
*S*_*j*_: the length of stay in the postoperative care unit for a patient who has type *j* surgery
 
*ts*: time to start surgery
 
*T*: number of time periods on the scheduling horizon
 
*U*^*p*^: the upper limit of resuscitation beds in the postoperative care unit
 
*λ*_*t*_: number of beds occupied from the previous scheduling cycle in the postoperative care unit at time t
 
*A*: number of surgeon assistants available to perform surgery
  Ω: maximum allowable delay in surgery
 
*Ô*_*j*_: the amount of time error expected for a type *j* surgery (in case of uncertainty)
  Γ: stable level value (in case of uncertainty)

### 3.3. Decision Variables

 
*Op*: number of extra beds in the postoperative care unit
 
*S*_*it*_: binary variable and equal to 1 if the patient *i* chooses a bed in the PACU at time *t*; 0 otherwise
 
*S*_*ht*_′: binary variable and equal to 1 if the emergency patient *h* occupies a bed in the PACU at time *t*; 0 otherwise
 
*X*_*irt*_: binary variable and equal to 1 if surgery is started at the beginning of time *t* for the selected patient *i* in operating room *r*; 0 otherwise
 
*X*_*hrt*_′: binary variable and equal to 1 if surgery is started at the beginning of time *t* for emergency patient *h* in operating room *r*; 0 otherwise
 
*y*_*irt*_: binary variable and equal to 1 if the selected patient *i* has a surgery at time *t* in the operating room *r*; 0 otherwise
 
*y*_*hrt*_′: binary variable and equal to 1 if the emergency patient *h* has a surgery at time *t* in the operating room *r*; 0 otherwise
 
*Q*_*iart*_: binary variable and equal to 1 if elective surgery *i* is assigned to surgeon a, operating room *r* and time *t*; 0 otherwise
 
*Q*_*hart*_′: binary variable and equal to 1 if emergency surgery *h* is assigned to surgeon a, operating room *r*, and time *t*; 0 otherwise
 
*Fa*: end time of last surgery of assistant surgeon *a*
 
*λ*: the dual variable corresponding to the uncertainty protection function

RETRACTED

### 3.4. Mathematical Modeling of the Problem

#### 3.4.1. Objective Function

(1) $$\begin{array}{c} \text{Min}Z1=\overset{I}{\underset{i=1}{\sum }}\overset{J}{\underset{j=1}{\sum }}\overset{R}{\underset{r=1}{\sum }}\overset{T+1}{\underset{t=t_{s}}{\sum }}\overset{T+1}{\underset{t^{\prime }=t_{s}}{\sum }}\left(1-g_{it}\right)*C_{jtt^{\prime }}*m_{ij}*X_{irt},\\ +\overset{H}{\underset{h=1}{\sum }}\overset{J}{\underset{j=1}{\sum }}\overset{R}{\underset{r=1}{\sum }}\overset{T+1}{\underset{t_{s}=1}{\sum }}r_{j}*m_{hj}^{\prime }*\left(1-X_{hrt_{s}}^{\prime }\right). \end{array}$$

Objective function (1) minimizes the cost of delay in elective surgeries and the cost of not accepting emergency surgeries.

(2) $$\begin{array}{c} \text{Max }Z2=\overset{I}{\underset{i=1}{\sum }}\overset{J}{\underset{j=1}{\sum }}\overset{R}{\underset{r=1}{\sum }}\overset{T+1}{\underset{t=t_{s}}{\sum }}m_{ij}*X_{irt}+\overset{H}{\underset{h=1}{\sum }}\overset{J}{\underset{j=1}{\sum }}\overset{R}{\underset{r=1}{\sum }}\overset{T+1}{\underset{t=t_{s}}{\sum }}m_{hj}^{\prime }*X_{hrt}^{\prime }. \end{array}$$

Objective function (2) maximizes the number of scheduled surgeries.

#### 3.4.2. Constraints

(3) $$\begin{array}{c} \overset{I}{\underset{i=1}{\sum }}X_{irt}+\overset{H}{\underset{h=1}{\sum }}X_{hrt}^{\prime }\leq 1\;;\forall r\;,\;t, \end{array}$$

(4) $$\begin{array}{c} \overset{I}{\underset{i=1}{\sum }}\overset{J}{\underset{j=1}{\sum }}m_{ij}*X_{irt}*O_{j}+\overset{H}{\underset{h=1}{\sum }}\overset{J}{\underset{j=1}{\sum }}m_{hj}^{\prime }*X_{hrt}^{\prime }*O_{j}\leq B_{rt}\;;\forall r\;,\;t, \end{array}$$

(5) $$\begin{array}{c} \overset{I}{\underset{i=1}{\sum }}\overset{J}{\underset{j=1}{\sum }}\overset{R}{\underset{r=1}{\sum }}m_{ij}*O_{j}*Q_{iart}+\overset{H}{\underset{h=1}{\sum }}\overset{J}{\underset{j=1}{\sum }}\overset{R}{\underset{r=1}{\sum }}m_{hj}^{\prime }*O_{j}*Q_{hart}^{\prime }\leq B_{at};\forall a\;,\;t, \end{array}$$

(6) $$\begin{array}{c} \overset{R}{\underset{r=1}{\sum }}\overset{T}{\underset{t=t_{s}}{\sum }}X_{irt}=1\;;\forall i, \end{array}$$

(7) $$\begin{array}{c} \overset{R}{\underset{r=1}{\sum }}X_{irt}\leq g_{it}\;;\forall i\;,\;t, \end{array}$$

(8) $$\begin{array}{c} \overset{R}{\underset{r=1}{\sum }}\overset{T}{\underset{t=t_{s}+1}{\sum }}X_{hrt}^{\prime }=0\;;\forall h, \end{array}$$

(9) $$\begin{array}{c} \overset{I}{\underset{i=1}{\sum }}\overset{R}{\underset{r=1}{\sum }}X_{irt}+\overset{H}{\underset{h=1}{\sum }}\overset{R}{\underset{r=1}{\sum }}X_{hrt}^{\prime }+\overset{I}{\underset{i=1}{\sum }}\overset{R}{\underset{r=1}{\sum }}y_{irt}+\overset{H}{\underset{h=1}{\sum }}\overset{R}{\underset{r=1}{\sum }}y_{hrt}^{\prime }\leq R;\forall t, \end{array}$$

(10) $$\begin{array}{c} \overset{I}{\underset{i=1}{\sum }}\overset{R}{\underset{r=1}{\sum }}X_{irt}+\overset{H}{\underset{h=1}{\sum }}\overset{R}{\underset{r=1}{\sum }}X_{hrt}^{\prime }+\overset{I}{\underset{i=1}{\sum }}\overset{R}{\underset{r=1}{\sum }}y_{irt}+\overset{H}{\underset{h=1}{\sum }}\overset{R}{\underset{r=1}{\sum }}y_{hrt}^{\prime }\leq A;\forall t, \end{array}$$

(11) $$\begin{array}{c} y_{irt^{\prime }}\geq m_{ij}*X_{irt};\forall i\;,\;j\;,\;r\;,\;t\;,t^{\prime }, \end{array}$$

(12) $$\begin{array}{c} y_{hrt\prime }^{\prime }\geq m_{hj}^{\prime }*X_{hrt}^{\prime };\forall h\;,\;j\;,\;r\;,\;t\;,t^{\prime }, \end{array}$$

(13) $$\begin{array}{c} s_{it^{\prime }}\geq \overset{R}{\underset{r=1}{\sum }}m_{ij}*X_{irt}\;;\forall i\;,\;r\;,\;t\;,t^{\prime }, \end{array}$$

(14) $$\begin{array}{c} s_{ht\prime }^{\prime }\geq \overset{R}{\underset{r=1}{\sum }}m_{hj}^{\prime }*X^{\prime }{}_{hrt}\;;\forall h\;,\;r\;,\;t\;,t^{\prime }, \end{array}$$

(15) $$\begin{array}{c} \overset{A}{\underset{a=1}{\sum }}Q_{iart}\geq m_{ij}*X_{irt}\;;\forall i\;,\;j\;,\;r\;,\;t\;, \end{array}$$

(16) $$\begin{array}{c} \overset{A}{\underset{a=1}{\sum }}Q_{hart}^{\prime }\geq m_{hj}^{\prime }*X_{hrt}^{\prime };\forall h\;,\;j\;,\;r\;,\;t\;, \end{array}$$

(17) $$\begin{array}{c} \overset{I}{\underset{i=1}{\sum }}s_{it}+\overset{H}{\underset{h=1}{\sum }}s_{ht}^{\prime }+\lambda_{t}\leq B^{p}+O^{p}\;;\forall t, \end{array}$$

(18) $$\begin{array}{c} O^{p}\leq U^{p}, \end{array}$$

(19) $$\begin{array}{c} F_{a}\geq \overset{I}{\underset{i=1}{\sum }}\overset{J}{\underset{j=1}{\sum }}\overset{R}{\underset{r=1}{\sum }}m_{ij}*O_{j}*Q_{iart}+\overset{H}{\underset{h=1}{\sum }}\overset{J}{\underset{j=1}{\sum }}\overset{R}{\underset{r=1}{\sum }}m_{hj}^{\prime }*O_{j}*Q_{hart}^{\prime };\forall a\;,\;t, \end{array}$$

(20) $$\begin{array}{c} X_{irt}\leq \overset{T}{\underset{t^{\prime }=t_{s}}{\sum }}X{'}_{hrt^{\prime }\;};\forall i\;,\;j\;,\;r\;,\;t, \end{array}$$

(21) $$\begin{array}{c} \overset{A}{\underset{a=1}{\sum }}\overset{R}{\underset{r=1}{\sum }}\overset{T}{\underset{t=t_{s}}{\sum }}Q_{iart}=1;\forall i, \end{array}$$

(22) $$\begin{array}{c} \overset{A}{\underset{a=1}{\sum }}\overset{R}{\underset{r=1}{\sum }}\overset{T}{\underset{t=t_{s}}{\sum }}Q_{hart}^{\prime }=1;\forall h, \end{array}$$

(23) $$\begin{array}{c} \overset{I}{\underset{i=1}{\sum }}Q_{iart}+\overset{H}{\underset{h=1}{\sum }}Q_{hart}^{\prime }\leq 1\;;\forall a\;,\;r\;,\;t\;, \end{array}$$

(24) $$\begin{array}{c} S_{it},X_{irt},y_{irt}\in \left\{0,1\right\};\forall i\;,\;r\;,\;t, \end{array}$$

(25) $$\begin{array}{c} S_{ht}^{\prime },X_{hrt}^{\prime },y_{hrt}^{\prime }\in \left\{0,1\right\};\forall h\;,\;r\;,\;t, \end{array}$$

(26) $$\begin{array}{c} O^{p}\geq 0\;an\;d\text{ integer,} \end{array}$$

(27) $$\begin{array}{c} Q_{iart}\in \left\{0,1\right\},Q_{hart}^{\prime }\in \left\{0,1\right\}. \end{array}$$

Equation (3) indicates that a maximum of one surgery can be performed in each operating room at any one time. Equation (4) states that the total time for elective and emergency surgeries should not exceed the total working time of each room. Equation (5) states that the total scheduled time for selective and emergency surgeries by each assistant surgeon should not exceed the total time available to the surgeon's assistant. Equation (6) allocates the start time to each surgery. Equation (7) prevents scheduling of selected surgeries between hours Ω from the current time *t*_*s*_ that have been rescheduled in the time window [*ts*, *ts* + Ω − 1].

RETRACTED

Equation (8) ensures that emergency surgeries are performed promptly. Equation (9) states that the total number of newly started and ongoing surgeries in each time period should not exceed the number of operating rooms. Limitation (10) states that the total number of surgeries performed in each time period should not exceed the number of surgeon assistants. Equations (11) and (12) determine the timing of each elective and emergency surgery. Equations (13) and (14) occupy beds in the PACU for a specified period of time indicate the patient of choice and emergency, respectively, until recovery from surgery. Equations (15) and (16) determine each elective and emergency surgery performance by the surgeon's assistant, respectively.

Equation (17) relates to PACU capacity. Equation (18) refers to the number of extra beds that can be added to the PACU according to rules, regulations, and space restrictions. Equation (19) determines the end time of the last surgery for each assistant surgeon. Equation (20) indicates the priority of surgery. Equations (21) and (22) relate to the appointment of an assistant surgeon. Equation (23) states that at any time, the number of surgeries performed simultaneously by each assistant surgeon cannot be more than one, and finally, equations (24)–(27) indicate the type of decision variables.

RETRACTED

### 3.5. Robust Optimization Model

Based on the available historical data, operating room managers provide an estimate of the time of each surgery according to its type, but since this parameter is affected by several factors, it is not predictable and cannot be considered definite values. Therefore, the model presented in this dissertation has uncertainty conditions in the parameter of expected time for surgery.

In this study, we discuss the function of Bertsimas and Sim [26] in the field of linear programming and discrete programming zero and one. In the model he presented for linear optimization, wire maintained the benefits of the linear framework proposed by Soyester [27], and the model he presented would provide an answer whose number of indefinite elements is determined by the analyst's discretion.

For example, linear programming with a Bertsimas and Sim's function becomes a robust linear programming model. In this function, one can have complete control over the degree of conservatism of any constraint using the Γ parameter.

We define the initial uncertain model assuming that only the elements of matrix A have uncertainty as follows:

(28) $$\begin{array}{c} \text{Min }C^{T}X,\\ \text{s.t}:\;\underset{j}{\sum }a_{ij}x_{j}-{\text{max}}_{\left|S_{i}\right|=\Gamma_{i}}\left\{\underset{j\in s_{i}}{\sum }{\hat{a}}_{ij}x_{j}\right\}\geq b_{i}\;;\forall i,\\ x\geq 0. \end{array}$$

The assumptions and definitions of the model components are as follows:

 
*S*_*i*_: a subset of coefficients in line *i* that have uncertainty.
 
${\hat{a}}_{ij}$: the value of the coefficient in line *i* where the jth coefficient has uncertainty (*j* ∈ *J*_*i*_)∈si, so that it changes in the interval.
  Γ_*i*_: adjustment of the robustness is the proposed method against the level of problem-solving conservatism. Each row has its own Γ_*i*_ parameter, which is not necessarily an integer and changes in the [0,|*J*_*i*_|] range.

In this case, the answer will be justified with a certain probability, which is described in detail in Bertsimas and Sim's dissertation. By obtaining the protection function and its linearization (the proof of relations is omitted), we will obtain the following robust model:

(29) $$\begin{array}{c} \text{Min }C^{T}X,\\ \text{s.t}:\;\underset{j}{\sum }a_{ij}x_{j}-\underset{j\in J_{i}}{\sum }p_{ij}-\lambda_{i}\Gamma_{i}\geq b_{i}\;;\;\forall i,\\ \lambda_{i}+p_{ij}\geq {\hat{a}}_{ij}x_{j}\;;\;\forall i,j\in J_{i},\\ p_{ij}\geq 0\;;\;\forall j\in J_{i},\\ \lambda_{i}\geq 0\;;\;\forall i,\\ x\geq 0. \end{array}$$

In interpreting the different values of gamma (degree of conservatism of the objective function) we will have: if the degree of conservatism of each row is equal to zero, then the model acts as a definite model, and if it takes its maximum value, it acts like the sweater approach with the maximum amount of conservatism. This parameter can also have values between these two.

RETRACTED

The robust optimization model will look like this after applying changes to limits that have an uncertainty parameter:

(30) $$\begin{array}{c} \text{Min }Z1=\overset{I}{\underset{i=1}{\sum }}\overset{J}{\underset{j=1}{\sum }}\overset{R}{\underset{r=1}{\sum }}\overset{T+1}{\underset{t=t_{s}}{\sum }}\overset{T+1}{\underset{t^{\prime }=t_{s}}{\sum }}\left(1-g_{it}\right)*C_{jtt^{\prime }}*m_{ij}*X_{irt},\\ +\overset{H}{\underset{h=1}{\sum }}\overset{J}{\underset{j=1}{\sum }}\overset{R}{\underset{r=1}{\sum }}\overset{T+1}{\underset{t_{s}=1}{\sum }}r_{j}*m_{hj}^{\prime }*\left(1-{Xhrt}_{s}^{\prime }\right),\\ \text{min }Z2=\overset{I}{\underset{i=1}{\sum }}\overset{J}{\underset{j=1}{\sum }}\overset{R}{\underset{r=1}{\sum }}\overset{T+1}{\underset{t=t_{s}}{\sum }}m_{ij}*X_{irt}+\overset{H}{\underset{h=1}{\sum }}\overset{J}{\underset{j=1}{\sum }}\overset{R}{\underset{r=1}{\sum }}\overset{T+1}{\underset{t=t_{s}}{\sum }}m_{hj}^{\prime }*X_{hrt}^{\prime }. \end{array}$$

Subject to Equations (1), (6)–(18), (20)–(27), and

(31) $$\begin{array}{c} \overset{I}{\underset{i=1}{\sum }}\overset{J}{\underset{j=1}{\sum }}m_{ij}*X_{irt}*{\text{Ō}}_{j}+\overset{J}{\underset{j=1}{\sum }}q1_{j}+\left(\lambda 1*\Gamma 1\right),\\ +\overset{H}{\underset{h=1}{\sum }}\overset{J}{\underset{j=1}{\sum }}m_{hj}^{\prime }*X_{hrt}^{\prime }*{\text{Ō}}_{j}+\overset{J}{\underset{j=1}{\sum }}q2_{j}+\left(\lambda 2*\Gamma 2\right)\leq B_{rt\;};\forall r\;,\;t,\\ q1_{j}+\lambda 1\geq \overset{I}{\underset{i=1}{\sum }}m_{ij}*X_{irt}*{\text{Ô}}_{j}\;;\forall j=1,\ldots ,J\;;\forall r\;,\;t,\\ q2_{j}+\lambda 2\geq \overset{H}{\underset{h=1}{\sum }}m_{hj}^{\prime }*X_{hrt}^{\prime }*{\text{Ô}}_{j}\;;\forall \;j\;,\;t,\\ q1_{j},\;\lambda 1,\;q2_{j},\;\lambda 2\geq 0,\\ \overset{I}{\underset{i=1}{\sum }}\overset{J}{\underset{j=1}{\sum }}\overset{R}{\underset{r=1}{\sum }}m_{ij}*{\text{Ō}}_{j}*Q_{iart}+\overset{J}{\underset{j=1}{\sum }}q3_{j}+\left(\lambda 3*\Gamma 3\right)\\ +\overset{H}{\underset{h=1}{\sum }}\overset{J}{\underset{j=1}{\sum }}\overset{R}{\underset{r=1}{\sum }}m_{hj}^{\prime }*{\text{Ō}}_{j}*Q_{hart}^{\prime }+\overset{J}{\underset{j=1}{\sum }}q4_{j}+\left(\lambda 4*\Gamma 4\right)\geq B_{at}\;;\forall \;a\;,\;t\\ q3_{j}+\lambda 3\geq \overset{I}{\underset{i=1}{\sum }}\overset{R}{\underset{r=1}{\sum }}m_{ij}*{\text{Ô}}_{j}*Q_{iart}\;;\forall \;j\;,\;a\;,\;t,\\ q4_{j}+\lambda 4\geq \overset{H}{\underset{h=1}{\sum }}\overset{R}{\underset{r=1}{\sum }}m_{hj}^{\prime }*{\text{Ô}}_{j}*Q_{hart}^{\prime }\;;\forall \;j\;,\;a\;,\;t,\\ q3_{j},\;\lambda 3,\;q4_{j},\;\lambda 4\geq 0,\\ F_{a}\geq \overset{I}{\underset{i=1}{\sum }}\overset{J}{\underset{j=1}{\sum }}\overset{R}{\underset{r=1}{\sum }}m_{ij}*{\text{Ō}}_{j}*Q_{iart}+\overset{J}{\underset{j=1}{\sum }}q5_{j}+\left(\lambda 5*\Gamma 5\right),\\ +\overset{H}{\underset{h=1}{\sum }}\overset{J}{\underset{j=1}{\sum }}\overset{R}{\underset{r=1}{\sum }}m_{hj}^{\prime }*{\text{Ō}}_{j}*Q_{hart}^{\prime }+\overset{J}{\underset{j=1}{\sum }}q6_{j}+\left(\lambda 6*\Gamma 6\right)\;;\forall \;a\;,\;t,\\ q5_{j}+\lambda 5\geq \overset{I}{\underset{i=1}{\sum }}\overset{R}{\underset{r=1}{\sum }}m_{ij}*{\text{Ô}}_{j}*Q_{iart}\;;\forall \;j\;,\;a\;,\;t,\\ q6_{j}+\lambda 6\geq \overset{H}{\underset{h=1}{\sum }}\overset{R}{\underset{r=1}{\sum }}m_{hj}^{\prime }*{\text{Ô}}_{j}*Q_{hart}^{\prime }\;;\forall \;j\;,\;a\;,\;t,\\ q5_{j},\;\lambda 5,\;q6_{j},\;\lambda 6\geq 0. \end{array}$$

RETRACTED

## 4. Gray Wolf Meta-Heuristic Algorithm

The gray wolf optimizer (GWO) algorithm is a nature-inspired meta-innovative algorithm that mimics the behavior of gray wolves and their leadership hierarchy and their hunting method. The gray wolf algorithm was proposed by Mirjalili et al. [1] based on their group hunting. The gray wolf is a member of the Canadian wolf family. Gray wolves are at the top of the food chain and prefer to live in groups. On average, their groups are 5–12. Interestingly, they have much stricter social governance. In this way, the alpha wolf is also called the ruling wolf in the group because his instructions must be followed by the group. Alphas are basically responsible for deciding on where to sleep, when to move, and so on.

The second level of grading of gray wolves is beta. Beta is alpha-controlled wolves that assist alpha in decision-making and other group activities. Beta wolf is probably the best candidate for an alpha, playing the role of a deputy for alpha and a moderator for the band. The lowest floor is the omega gray wolf. Omega wolves play the role of victims for other members of the group. They are the last wolves allowed to eat. If the wolf is not alpha, beta, or omega, he is called obedient (or delta). Delta wolves follow alpha and beta and rule occasionally. To mathematically model the social governance of wolves, the most appropriate solution is called wolves [23, 24].

RETRACTED

As a result, the second and third better solutions were named wolf *β* and *δ*, respectively. The remaining solutions are assumed to be *ω*. Therefore, in the GWO algorithm, optimization is guided by *δ*,*β* and *α* and *ω* wolves follow these three categories. Gray wolves bypass prey during hunting. For mathematical modeling, the circumvention of equations (32) and (33) has been proposed [25].

(32) $$\begin{array}{c} \overset{⟶}{D}=\left|\overset{⟶}{C}.\overset{⟶}{X_{P}}\left(t\right)-\overset{⟶}{X}\left(t\right)\right|, \end{array}$$

(33) $$\begin{array}{c} \overset{⟶}{X}\left(t+1\right)=X_{P}\left(t\right)-\overset{⟶}{A}.\overset{⟶}{D}, \end{array}$$

where *t* represents the flow repetition, *A* and *C* represent the vector coefficient and the hunting position vector, and *X* represents the position vector of a gray wolf. Vectors *A* and *C* are calculated according to the following equations:

(34) $$\begin{array}{c} \overset{⟶}{A}=2\overset{⟶}{a}.\overset{⟶}{r_{1}}-\overset{⟶}{a}, \end{array}$$

(35) $$\begin{array}{c} \overset{⟶}{C}=2.\overset{⟶}{r_{2}}. \end{array}$$

We have that the $\overset{⟶}{a}$ elements are reduced linearly from 2 to 0 under the iteration path, and *r*1 and *r*2 are the random vectors in the range [0, 1] [28].

Gray wolves have the ability to detect the position of prey and bypass them. Hunting is usually guided by alpha. Beta and delta may also occasionally participate in hunting. Therefore, in an absolute search space, we have no solution for the optimal position (hunting). To mathematically simulate the hunting behavior of gray wolves, we assume that alpha (candidate best solution), beta, and delta are sufficiently aware of the potential hunting position. We need to force the other search agents to update their position according to the position of the best search agents. This operation is performed according to the following equations:

(36) $$\begin{array}{c} \overset{⟶}{D_{\alpha }}=\left|\overset{⟶}{C_{1}}.\overset{⟶}{X_{\alpha }}-\overset{⟶}{X}\right|,\\ \overset{⟶}{D_{\beta }}=\left|\overset{⟶}{C_{2}}.\overset{⟶}{X_{\beta }}-\overset{⟶}{X}\right|,\\ \overset{⟶}{D_{\delta }}=\left|\overset{⟶}{C_{3}}.\overset{⟶}{X_{\delta }}-\overset{⟶}{X}\right|, \end{array}$$

(37) $$\begin{array}{c} {\overset{⟶}{X}}_{1}=\overset{⟶}{X_{\alpha }}-\overset{⟶}{A_{1}}.\left({\overset{⟶}{D}}_{\alpha }\right),\\ {\overset{⟶}{X}}_{2}=\overset{⟶}{X_{\beta }}-\overset{⟶}{A_{1}}.\left({\overset{⟶}{D}}_{\beta }\right),\\ {\overset{⟶}{X}}_{3}=\overset{⟶}{X_{\delta }}-\overset{⟶}{A_{1}}.\left({\overset{⟶}{D}}_{\delta }\right), \end{array}$$

(38) $$\begin{array}{c} \overset{⟶}{X}\left(t+1\right)=\frac{{\overset{⟶}{X}}_{1}+{\overset{⟶}{X}}_{2}+{\overset{⟶}{X}}_{3}}{3}. \end{array}$$

In short, in the GWO algorithm, the search process begins with the creation of a random population of gray wolves (candidate solutions). During the iteration period, alpha, beta, and delta wolves estimate the probable hunting position. Each candidate solution updates its distance with the bait. Parameter *A* is reduced from 2 to 0 to enhance the detection and attack process. When |*A*| > 1, the candidate solutions diverge, and when |*A*| < 1, the candidate solutions converge.

RETRACTED

## 5. Results

This section analyzes the proposed model and its results. To evaluate the efficiency of the proposed model, one of the Asian hospitals is studied. In order to validate the proposed model for the definite and solid problem, GAMS 24.0 software and CPLEX method are used, and the solution results are analyzed in the certain and robust model, and then, we will provide the sensitivity analysis of the basic parameters of the model.

According to Tables 1 and 2, emergency surgeries are scheduled for the first time due to their high priority over other surgeries, and selective surgeries are scheduled for other time periods. The planning of the operating room where each surgery should be performed is also shown in Table 1. In Table 2, in addition to scheduling surgeries, the surgical assistant who must be present to perform each surgery is also scheduled. As it is known, due to the limitation of the number of operating rooms, it is possible to perform four surgeries at the same time, so in each part of the time, four surgeons are working.

Figures 1 and 2 show the first objective function considering the uncertainty coefficient of 0.05, 0.1, 0.25, and 0.5. As it turns out, the amount of costs increases with increasing uncertainty. On the other hand, by constantly considering the number of selected patients, costs decrease with an increasing number of emergency patients (Figure 1), and also by constantly considering the number of emergency patients, costs increase with an increasing number of selected patients (Figure 2). This may be due to the fact that the selected patients have more surgical transfers than the program envisaged by the management, which incurs costs.

### 5.1. Evaluation of the Efficiency of the Proposed Solution Method

Endoscopic surgery is not considered in this study. There are 12 residents and 2 fellowships in this hospital, which have the ability to perform certain operations depending on the academic year and the experience gained. In addition to the surgeon, each surgery requires a team of technicians (anesthesiologist, anesthesiologist, and operating room technician). In some surgeries, in addition to the surgeon, the surgeon's help is also needed. There is a recovery bed as well as medical equipment related to each type of operation.

RETRACTED

In that study, data from all operations performed in operating rooms over two years were collected from a hospital database. These data include a list of patients at each date, operation code, operation name, start and end time of operation, name of the surgeon, and assistant surgeon. Some of the information was also collected from experts is as follows:

- Surgeon data: the surgeries that each surgeon is able to perform, the residents' training program (including the operations they must perform in each course), the operations that each surgeon can perform
- Equipment related: types of equipment available and their inventory, type, and number of equipment used for each operation
- Surgery related: types of surgery (urology, laparoscope, etc.), surgeries that require the help of a surgeon
- Operating room related: the number of operating rooms, rooms equipped with special equipment, surgeries that can be performed in each room
- Technician groups related: the number of technician groups in each shift per day

Using the collected data and frequency graphs and the duration of different operations, the discrete probability distribution of the duration of each type of operation has been approximated. The time distribution of different operations is completely different.

Actual data from the 15 days of the study hospital were used to evaluate the proposed approach. The information for each issue is information about the actual day of surgery of the hospital. This information includes a list of surgeries per day, type of surgery, possible surgeons for each surgery, number of operating rooms available, number of technicians available, number of beds in the preoperative and recovery wards, equipment needed for each surgery, the available number of equipment, and the surgeon's assistants are possible for each operation.

For the duration of the surgeries in the definite case, the average time of the surgeries is used, and for the probable case, the probability distribution function of the times of each surgery is used.

First, the problem is solved by considering the average duration of surgery in the definite case using the gray wolf algorithm. In this algorithm, the number of wolves per repetition is equal to 10, and the condition for stopping the algorithm from achieving a better answer in 100 consecutive repetitions, the position change coefficient equal to 0.03, the impact factor of the best position of each wolf equal to 1, and the impact factor of the wolf community equal to 3 are considered. The parameters of the algorithm are set by running the algorithm on a sample of different problems and using the method of simultaneous tuning of the parameters by using self-organizing neural networks.

RETRACTED

To select the most effective innovative information in the design of the GWO algorithm, the following seven scenarios have been designed:

  Scenario 1: selection of the next surgery as well as allocation of resources to each stage of the surgery. It should be done without considering the innovative information and only based on the amount of pheromone.
  Scenario 2: the first level of innovative information is based on LPT, and the second level of innovative information is based on ES.
  Scenario 3: level 1 of innovative information based on LPT and level 2 of innovative information for surgeon selection based on LFM and for other sources based on ES.
  Scenario 4: the first level of innovative information is based on LFJ, and the second level of innovative information is based on ES.
  Scenario 5: initiative information of the first level for the first surgery is based on LFJ and for other surgeries is based on LPT, and innovative information of the second level is to select the surgeon of the first surgery based on LFM and for other surgeries based on ES.
  Scenario 6: initial level 1 information for selecting the first two surgeries based on LFJ and for other surgeries based on LPT, and innovative level 2 information for selecting the surgeon for the first two surgeries based on LFM and for other surgeries based on ES.
  Scenario 7: level 1 of innovative information based on LFJ and level 2 innovative information for surgeon selection based on LFM and for other sources based on ES.

The data for the 15 actual samples are given in Table 3. Each instance is solved in 10 replications, and the mean of the objective function under different scenarios is given in Table 3.

In this research, the performance of the GWO algorithm for optimizing the robust model with the optimal solution of the mathematical model and the answer obtained from the algorithm of Xiang et al. The authors of [5] designed to test the performance of the GWO algorithm, the answer obtained from this algorithm in the definite state in 15 real problem samples with the optimal definite problem solution obtained from solving the mathematical programming model in GAMS software and the answer obtained are compared by the algorithm of Xiang et al.

Designed to test the performance of the GWO algorithm, the answer obtained from this algorithm in the definite state in 15 real problem samples with the optimal definite problem solution obtained from solving the mathematical programming model in GAMS software and the answer obtained are compared by the algorithm of Xiang et al. [5].

RETRACTED

Table 4 shows the impact of using innovative rules in the design of the GWO algorithm. The numbers in the first column of this table indicate the state of nonuse of innovative information, which is significantly higher than the numbers in the other columns. The following columns each show the different combinations of considered innovative rules. The results of Table 4 show that Scenario 7 has the lowest rates of overtime and unemployment; Scenario 7 is therefore used in the design of the GWO algorithm. It also compares the best solution obtained from the GWO method with the optimal solution obtained from the mathematical programming model of the problem in the definite case and the solution obtained from the algorithm of Xiang et al. [5].

Comparison of GWO results with optimal solutions proves the efficiency of the proposed algorithm. Out of 15 cases, the algorithm has reached the optimal solution in 13 cases and is slightly different from the optimal solution in 2 cases; also, the results of comparing the proposed algorithm with the algorithm of Xiang et al. [5] show the superiority of the designed GWO algorithm. In all cases, both algorithms have the same solutions, or the solution of the algorithm designed in this research is significantly better.

To better show the results of different methods in the definite case, a sample problem with 19 surgeries and 4 operating rooms was solved with different methods and Gantt diagram of the results of the GWO algorithm of Xiang et al. [5], GWO was designed in this study, and the results of the solid mathematical model are depicted in Figures 3 and 4. The numbers shown in each rectangle in these diagrams represent the code for each surgery.

According to Figure 3, in solving this sample problem with Xiang et al.'s [5] algorithm, operating room 3 has two unemployment time blocks between surgeries, which is due to sharing the surgeon's source in surgeries 121 and 122. This means that both surgeries 121 and 122 are assigned to surgeon number 1. On the other hand, as Figure 3 shows, due to the unbalanced distribution of operations in different rooms, overwork occurred in operating room 2. In operating room 3, however, there is an unused time period.  Figure 4 shows the Gantt diagram of the results of the GWO algorithm proposed in this study and the results of the certain optimal model.

Figure 4 shows that although the two proposed GWO methods and the definitive model lead to different answers, they do not differ in the value of the objective function, which shows the efficiency of the proposed GWO algorithm.

After confirming the performance of the designed GWO in the final state, this section evaluates the simulation-based optimization (GWO simulation); for this purpose, 15 real problems have been solved using this algorithm in terms of the probability of the duration of surgery. Table 4 shows the results of solving each problem in 100 iterations of the simulation.

RETRACTED

For each problem, the answers obtained (including the sequence of surgeries and the allocation of resources to each stage) are tested on the following scenarios, and the results are presented in Table 5:

  Scenario 1: longest surgery scenario; in this scenario, it is assumed that all surgeries are at their maximum time, and the goal is to obtain the objective function in the worst case.
  Scenario 2: average value scenario; in this scenario, the time of surgery is equal to the average value.
  Scenario 3: the shortest surgical time scenario; in this scenario, it is assumed that all surgeries are in their shortest time. The goal is to obtain the objective function at its best.

Table 5 shows the worst, best, and mediocre results that can be obtained for the answer obtained from the GWO in each of the problems. In order to validate the GWO simulation method, the criterion of using the probabilistic model (VSS) 1 has been used. VSS is the value of considering uncertainty by determining the value of the optimal objective function of the probability problem and the expected value of the objective function for the optimal solution of the problem of the mean value [1, 5, 27–34].

The mean value problem is the definite problem equivalent to the problem considering the average duration of each action. In other words, this value indicates the value of using the probabilistic model instead of the definitive model. To determine the value of the GWO simulation method in comparison with the GWO algorithm, the solution of the combined simulation-based optimization method with the answer obtained from the GWO algorithm for the mean value of the operation time is compared in conditions of uncertainty. For this purpose, for each sample of the problem, the answer to the problem is first obtained by considering the average duration of surgery with the GWO algorithm. In these samples, the average duration of the operation is considered for each surgery. In this experiment, examples of problems are considered that the GWO algorithm has finally achieved the optimal solution. Each answer includes the sequence of surgeries, and how resources are allocated to them; then, for the same example of problems, the solution of the problem is obtained by implementing a hybrid optimization algorithm based on simulation and considering uncertain conditions.

In order to compare the results of these two methods, for each problem sample, 50 test scenarios with random numbers were created from the probability function of the duration of surgery; each scenario shows a possible combination of the duration of the surgery. The solutions of the two-level GWO algorithm (including the sequence of surgeries and resource allocation) and the answers of the GWO algorithm based on simulation (GWO simulation) are related to 12 problems, run with these scenarios, and for each test problem, the average value of the objective function is 50. The scenario is calculated. The results of comparing the mean of the objective function in the scenarios for the answers of the GWO algorithm and the hybrid algorithm are shown in Table 6.

RETRACTED

The results presented in Table 6 show that in conditions of uncertainty, the answers obtained by the GWO simulation method are in all cases better than the answers obtained by the GWO algorithm. And only in one case with a slight difference is the GWO answer better. The analysis of the results shows that in conditions of uncertainty, the answers obtained by the GWO simulation method are on average 73.75% better than the answers obtained by the GWO algorithm. The comparison results of the GWO simulation method and GWO algorithm are shown in Figure 5.

Figure 5 clearly shows the superiority of the proposed hybrid method compared to the GWO algorithm. Although GWO simulation has been tested on problems the size of the actual problems of the studded hospital, this algorithm is also capable of solving larger test problems.

## 6. Conclusion

The field of health has received much attention in recent years, and given the importance of operating rooms and the costs of this part of the hospital, the timing of operating rooms is very important. Therefore, in this article, the issue of operating room scheduling has been studied by considering some existing conditions and limitations.

Considering the operating room separately does not fully address the actual conditions and features of the operating room planning and scheduling issue. Therefore, in this article, several operating rooms and types of surgeries are considered. Also, the operating room and resuscitation sections are considered as two sections that affect each other and are closely related to each other.

Patients who apply for surgery have different priorities according to the type of surgery and degree of sensitivity. The main effect of considering the priority of patients in the context of social services is seen during the time each patient waits for surgery, and patients with more sensitive surgery have a higher priority for surgery. In addition to the operating room time restrictions, the capacity of the resuscitation ward is also limited in terms of the number of beds available and the duration of the patient's stay in the unit.

RETRACTED

One of the most important factors in the complexity of patients' planning and scheduling issues is the uncertainty in the duration of surgeries because this factor is influenced by many factors and even in similar surgeries due to certain patient conditions, and the need to use special tools and the duration of surgery are not the same. Also, the presence of a surgeon's assistant in any surgery can improve the outcome of surgery in cases such as reducing the time of surgery and reducing the possibility of errors and mistakes in surgery.

According to the hypotheses and cases mentioned, a multiobjective mathematical planning model for the operating room scheduling problem is presented, and a case study has been conducted in one of the hospitals in East Asia. The LP-metric method for solving the selected model, as well as the uncertainty in the surgical time parameter, has been investigated, and the model solution results for the problem with different dimensions are presented. The GWO algorithm is also used to solve the model in large dimensions. Due to the uncertainty in the problem under study, this algorithm was combined with the simulation approach, and a new method called GWO simulation was proposed. The results show that with increasing the stability factor in the problem state, the value of the objective function also increases, which indicates that as the model stability increases, the operating room will incur more costs. In other words, the more resistant we are to the answer to uncertainty, the more we have to pay to find the optimal answer. The proposed meta-heuristic algorithm can also be used as a new and efficient tool in operating room scheduling in emergencies.

## Figures and Tables

**Figure 1:** Results of the first objective function for *I* = 10 and for *H* = 1 and *H* = 2 under uncertainty.

**Figure 2:** Results of the first objective function for *H* = 3 and for *I* = 15 and *I* = 24 under uncertainty.

**Figure 3:** Gantt chart of Xiang et al.'s [5] results in solving a sample problem.

**Figure 4:** Gantt chart of the results of the GWO algorithm proposed in this study in solving the sample problem.

**Figure 5:** Comparison of the GWO with the GWO simulation.

**Table 1:** Optimal solution of operation room scheduling.

	T1	T2	T3	T4	T5	T6	T7	T8
R1	H2	I14	I3		I20	I8	I13	I11
R2	H3	I7	I2	I15	I21	I6	I23	I5
R3	H1	I9	I25	I19	I10	I22	I24	I1
R4	H4	I16	I18		I4		I12	I17

**Table 2:** Optimal solution of surgical assistant scheduling.

	T1	T2	T3	T4	T5	T6	T7	T8
A1	H3		I25					I11
A2		I14	I18					
A3					I10			
A4		I9				I6	I24	I17
A5		I7	I2				I12	I5
A6	H4	I16			I21	I22		
A7	H1			I19	I4		I23	
A8	H2		I3	I15	I20	I8	I13	I1

RETRACTED

**Table 3:** Results of different scenarios of different combinations of innovative rules in GWO algorithm design.

Test problem	Number of surgeries	Number of surgeons	Number of operating rooms	Average objective value						
				Scenario 1	Scenario 2	Scenario 3	Scenario 4	Scenario 5	Scenario 6	Scenario 7
1	16	9	6	4.32	4.11	2.05	0.68	0.22	0.00	0.00
2	23	11	7	53.87	57.83	43.11	49.56	0.22	3.31	0.00
3	27	12	7	141.16	29.11	29.16	34.53	19.87	23.47	0.00
4	22	10	7	7.19	0.92	3.87	0.00	0.49	2.37	0.00
5	16	12	7	0.00	0.26	0.00	0.00	0.00	0.00	0.00
6	27	9	7	47.16	3.48	5.68	2.97	2.47	3.83	0.00
7	25	9	7	94.18	78.15	84.19	104.35	23.19	20.04	0.00
8	18	11	7	2.41	0.00	0.00	0.00	0.00	0.00	0.00
9	18	9	7	57.19	20.19	74.83	34.86	0.00	0.25	0.00
10	22	11	7	84.19	32.87	37.89	39.96	34.18	32.73	27.92
11	21	8	7	16.79	1.98	7.88	2.64	2.54	1.44	0.00
12	17	9	7	4.53	0.00	0.00	0.81	0.00	0.00	0.00
13	20	16	8	5.79	16.23	6.75	0.00	0.00	0.00	0.00
14	22	12	7	3.72	0.25	0.00	0.00	0.00	0.00	0.00
15	19	9	8	26.93	20.19	37.14	18.92	3.19	2.19	0.00
Average				36.63	17.70	22.17	19.29	5.76	5.98	1.86

**Table 4:** Results of the proposed hybrid algorithm in the sample of different problems.

Test problem	Number of surgeries	Number of surgeons	Number of operating rooms	Average objective value	CPU time
1	16	9	6	0.18	2
2	23	11	7	3.85	11
3	27	12	7	25.36	37
4	22	10	7	0.00	20
5	16	12	7	0.00	1
6	27	9	7	5.08	27
7	25	9	7	5.81	16
8	18	11	7	2.63	5
9	18	9	7	0.00	1
10	22	11	7	41.04	26
11	21	8	7	0.95	18
12	17	9	7	0.00	1
13	20	16	8	0.00	1
14	22	12	7	0.09	31
15	19	9	8	0.00	17

**Table 5:** Evaluation of GWO simulation response on different scenarios.

Number of solutions	Number of surgeries	Worst scenario			Average value scenario			Best scenario		
		Overtime	Idle time	Objective value	Overtime	Idle time	Objective value	Overtime	Idle time	Objective value
1	14	0	4	9.12	0	0	0	0	0	0
2	19	6	0	26.46	0	0	0	0	0	0
3	223	19	5	11.28	2	2	9.38	0	0	0
4	21	19	0	7.29	0	0	0	0	0	0
5	14	0	0	0	0	0	0	0	0	0
6	25	11	2	42.59	3	0	14.75	0	0	0
7	23	9	0	37.25	3	5	16.86	0	0	0
8	16	2	0	5.39	0	0	0	0	0	0
9	19	0	0	0	0	0	0	0	0	0
10	21	42	0	18.93	12	0	47.39	0	0	0
11	19	0	0	0	0	0	0	0	0	0
12	15	0	0	0	0	0	0	0	0	0
13	18	0	0	0	0	0	0	0	0	0
14	24	9	5	26.43	0	0	0	0	0	0
15	17	0	3	5.69	0	0	0	0	0	0

**Table 6:** Comparison of the proposed hybrid method (GWO simulation) and pure GWO algorithm.

Test problem	Number of surgeries	Number of surgeons	Number of operating rooms	Average GWO objective function in scenarios	Mean GWO simulation objective function in scenarios	Percentage of improvement in average responses (VSS)
1	15	6	5	21.452	5.492	73.3
2	20	9	5	6.957	0	100
3	25	10	5	12.79	3.482	74.28
4	20	8	5	3.752	0	100
5	15	10	5	59.73	4.483	95.79
6	25	7	5	9.672	1.572	78.27
7	24	7	5	0.728	0.947	0
8	18	9	5	2.783	0	100
9	16	7	5	1.466	0.792	46.37
10	20	9	4	2.886	0.591	78.42
11	19	6	4	8.394	1.924	76.92
12	15	5	4	1.067	0.219	97.68
Average improvement (percentage)						73.75

RETRACTED

## Data Availability

The data underlying the results presented in the study are available within the manuscript.
